# Targeted Knockdown of IQGAP1 Inhibits the Progression of Esophageal Squamous Cell Carcinoma *In Vitro* and *In Vivo*

**DOI:** 10.1371/journal.pone.0096501

**Published:** 2014-05-06

**Authors:** Xiao-Xia Wang, Kang Wang, Xiao-Zhong Li, Li-Qin Zhai, Chong-Xiao Qu, Yan Zhao, Zhi-Rong Liu, Hui-Zhen Wang, Qi-Jun An, Li-Wei Jing, Xu-Hong Wang

**Affiliations:** 1 Department of Biochemistry and Molecular Biology, Shanxi Medical University, Taiyuan, China; 2 Department of Emergency, Shanxi Provincial People's Hospital, Taiyuan, China; 3 Department of Pathology, Shanxi Provincial People's Hospital, Taiyuan, China; 4 Department of Statistics, Shanxi Medical University, Taiyuan, China; 5 Department of Surgery, Shanxi Cancer Hospital, Taiyuan, China; Vanderbilt University, United States of America

## Abstract

IQGAP1 is a scaffolding protein that can regulate several distinct signaling pathways. The accumulating evidence has demonstrated that IQGAP1 plays an important role in tumorigenesis and tumor progression. However, the function of IQGAP1 in esophageal squamous cell carcinoma (ESCC) has not been thoroughly investigated. In the present study, we showed that IQGAP1 was overexpressed in ESCC tumor tissues, and its overexpression was correlated with the invasion depth of ESCC. Importantly, by using RNA interference (RNAi) technology we successfully silenced IQGAP1 gene in two ESCC cell lines, EC9706 and KYSE150, and for the first time found that suppressing IQGAP1 expression not only obviously reduced the tumor cell growth, migration and invasion *in vitro* but also markedly inhibited the tumor growth, invasion, lymph node and lung metastasis in xenograft mice. Furthermore, Knockdown of IQGAP1 expression in ESCC cell lines led to a reversion of epithelial to mesenchymal transition (EMT) progress. These results suggest that IQGAP1 plays crucial roles in regulating ESCC occurrence and progression. IQGAP1 silencing may therefore develop into a promising novel anticancer therapy.

## Introduction

Esophageal squamous cell carcinoma (ESCC) is one of the most aggressive carcinomas of the gastrointestinal tract in the world, with a particularly high incidence rate in China [1], [2]. Despite rapid advances in surgery, chemotherapy, and radiotherapy, the prognosis of ESCC patients has not significantly improved [3]. In order to develop more effective diagnosis and therapeutic technologies, it is important to obtain a better understanding of the genetic alterations responsible for the molecular biological changes associated with human ESCC development and progression.

IQGAP1 (IQ-domain GTPase-activating protein 1) is a scaffolding protein that contains multiple protein-interacting domains [4]–[6]. Through binding to various proteins, IQGAP1 regulates various basic cellular activities, such as cell-cell adhesion [7], cytoskeletal regulation [8], [9], directional migration and transcription [7], [10]–[13]. Importantly, accumulating evidence has demonstrated that IQGAP1 plays an important role in tumorigenesis and tumor progression. It has been shown that IQGAP1 is upregulated in various tumor types, including colorectal carcinoma [14], [15], gastric cancer [16], [17] and hepatocellular carcinoma [18], [19]. Recently, we have found that IQGAP1 is overexpressed in pancreatic cancer [20]. Moreover, IQGAP1 overexpression and diffuse invasion pattern are associated with poor prognosis in ovarian carcinomas and colorectal carcinoma [14], [21]. These findings thus provide compelling evidence that IQGAP1 plays an important role in tumor development and progression. However, the roles of IQGAP1in ESCC remain unclear.

In the present study, we first detected IQGAP1 expression in ESCC tumor tissues compared with the matched adjacent normal tissues and its relationship with clinicopathological features. Then, we investigated the effects of IQGAP1 knockdown on ESCC cell growth, invasion and metastasis *in vitro* and *in vivo*. Moreover, we observed the effects of IQGAP1 knockdown on the regulation of epithelial and mesenchymal markers.

## Materials and Methods

### Ethics Statement

This study was conducted in accordance with the Helsinki declaration. All the patients gave their written informed consent to participate in the study. The study was approved by the Research Ethics Committee at Shanxi Medical University.

The animal experimental protocol was approved by the Animal Care and Use Committee of Shanxi Medical University.

### Tissue samples

Seventy-five patients with ESCC diagnosed were selected from the formalin-fixed paraffin embedded archives of the Shanghai Biochip Company. All samples were analyzed in a tissue microarray (TMA) format which was constructed with a Beecher Instruments Tissue Array (Silver Spring, MD) as described previously [20]. In addition, fresh tissue samples of 4 ESCC were collected from Shanxi Cancer Hospital. The corresponding normal esophageal epithelium was taken from the matched distal resected margin of ESCC samples which was tumor-free. All surgical specimens were separated by experienced pathologists and proved by histopathologic examination. Fresh samples were dissected manually to remove connective tissues and stored in liquid nitrogen immediately until further use. The patients received no radiotherapy or chemotherapy before surgery.

### Immunohistochemical analysis

Immunohistochemical analysis was performed as mentioned before [20]. The slides were evaluated for immunostaining independently by two investigators who were blinded to clinicopathologic data. Each sample was assigned by the extent of immunoreactivity to one of the following categories: 0 (0–4%), 1 (5–24%), 2 (25–49%), 3 (50–74%) or 4 (75–100%). The intensity of immunostaining was determined as 0 (negative), 1+ (weak), 2+ (moderate) or 3+ (strong). A final immunoreactivity score of each section was obtained by multiplying the two individual scores and was divided into four levels: ‘0’, negative; ‘1∼4’, weak; ‘5∼8’, moderate; ‘9∼12’, strong. Score 0 to 4 was regarded as negative expression, and score 5 to 12 was regarded as positive expression.

### Western blot

Whole cell extracts were prepared from ESCC and adjacent normal tissues and cultured cells by homogenizing cells in a lysis buffer [10 mM Tris-HCl (pH 7.5), 150 mM NaCl, 2 mM ethylenediaminetetraacetic acid (EDTA), 1% Triton X-100] containing a cocktail of protease inhibitors. The supernatant was collected after centrifugation at 12 000 g for 15 min, and subjected to Western blot as previously described [20]. The anti-IQGAP1 (1∶5000), anti-E-cadherin (1∶500) and anti-N-cadherin (1∶500) antibodies were purchased from BD Biosciences. The anti-cyclin D1 (1∶500), anti-cyclin B1 (1∶1000), anti-CDK1 (1∶1000) and anti-CDK4 (1∶500) antibodies were purchased from ABclonal Biotechnology. Densitometry was performed by Kodak Molecular Imaging Software.

### Reverse transcription-PCR (RT-PCR)

Total RNA was extracted from tissues and cultured cells by using the Trizol reagent (Invitrogen) following the manufacturer's instructions. Purified RNA was reverse transcribed to the first strand of cDNA primed with random hexamers using SuperScript First-Strand Synthesis System for RT-PCR kit (Invitrogen). PCR was then performed at annealing temperature of 58°C for 30 cycles with cDNA as template. The primers were as follows: forward primer 5′-GGAGCACAATGATCCAATCC-3′ and reverse primer 5′-ATGGTTCGA GCATCCATTTC-3′ for IQGAP1 gene. Forward primer 5′-GGCCTCCAA GGAGTAAGACC-3′ and reverse primer 5′-AGGGGTCTACATGGCAACTG-3′ for GAPDH (glyceraldehyde-3 -phosphate dehydrogenase) gene.

### Cell culture and stable cell line selection

Human ESCC cell line EC9706 and KYSE150 were obtained from the Tumor Cell Bank of Chinese Academy of Medical Science and normal esophageal cell line Het-1A was obtained from the Cell Bank of Shanghai Bioleaf (China). The cells were cultured in RPMI 1640 medium with 10% fetal bovine serum (FBS). The EC9706 and KYSE150 cells were plated into six-well plates for 24 h and then transfected with IQGAP1 RNA interference (RNAi) plasmid using LipofectAMINE 2000 (Invitrogen) according to the manufacturer's instruction. The sequence of the IQGAP1 siRNA used in this study is as follows: 5'-CAACGACATTGCCAGGGATAT-3'. 24 h after transfection, the cells were split at ratios of 1∶10 and stable transfectants were selected in G418 at a concentration of 400 mg/L. Thereafter, the selection medium was replaced every 3 days. After 2 weeks of selection in G418, clones of resistant cells were isolated and then further subcloned by serial dilution to establish single cell clones. The stable IQGAP1 RNAi clones were expanded and used for the following studies.

### Cell proliferation assay

Cells were seeded into 96-well culture plates for 0–10 days. Cell proliferation was determined by adding 5 mg/ml MTT [3-(4, 5-dimethylthiazol-2-yl)-2, 5-diphenyltrazolium bromide] and incubating the cells further for 4 h, then 150 µl DMSO was pipetted to solubilize the dark blue formazan product for 10 min. Absorbance at a wavelength of 570 nm in each well was measured using an automated microplate reader (Bio-Rad, Hercules).

### Colony formation assay

Cells were plated on 100 mm plates and cultured for 14 days. The colonies were stained with 0.1% crystal violet after fixation with 4% formaldehyde. The positive colony formation was counted under a microscopic field (×100).

### Cell cycle analysis

The cells were harvested, washed once in phosphate-buffered saline (PBS) and fixed in 70% ethanol for 24 h. Staining for DNA content was performed with 50 mg/ml propidium iodide and 1 mg/ml RNase A for 30 min at room temperature. Data were collected using BD Calibur flow cytometer.

### Wound healing assay

Cells were grown to confluence and then wounded using a 200-µl pipet tip. Plates were washed with PBS to remove detached cells and incubated with RPMI 1640 medium without FBS. Images of the wounds were taken immediately (0 h) and 48 h, respectively. The motility speed of cells was assessed by the healing degree of the wound line.

### *In vitro* migration and invasion assays

For transwell chamber-based motility and invasion assays, 30 ul RPMI1640 medium was added to the lower chambers, 2×10^4^ cells/well were added to the upper chambers and allowed to pass through an 8-µm-pore polycarbonate filter, which had been either pre-coated with 1 mg/ml Matrigel (BD Biosciences) for invasion assay or uncoated for migration assay. Nonmigrating cells on the upper surface were carefully removed with a cotton swab. The filters were then fixed in methanol, stained with 0.1% crystal violet and counted under a microscope (×100).

### Xenograft assays in nude mice

Male BALB/c nu/nu mice (4–6 weeks old) were purchased from Vital River Laboratory Animal Technology Co. Ltd (Beijing, China). 1×10^6^ cells in 0.1 ml of PBS were inoculated subcutaneously (s.c.) into nude mice (six for each group). The tumor volume (cm^3^) was calculated according to the following formula: length × width^2^/2. The mice were sacrificed 12 weeks after injection and examined for s.c. tumor growth and metastasis development. The tissues were embedded in paraffin and stained with hematoxylin and eosin (H&E).

### Immunofluorescence

Cells grown on coverslips were fixed with cold methanol for 30 min. Then, the cells were washed with PBS and incubated with anti-IQGAP1 (1∶200), anti-E-cadherin (1∶100), or anti- N-cadherin (1∶100) antibodies overnight at 4°C. The cells were then washed with PBS and incubated with TRITC-conjugated secondary antibodies (Zhongshan Golden Bridge) for 30 min. Nuclei were counter stained with 4′,6-diamino-2-phenylindole (DAPI; Invitrogen). The images were obtained using a fluorescence microscope (BX50; Olympus, Inc., Tokyo, Japan).

### Statistical analysis

All statistical analyses were carried out using the SPSS 16.0 statistical software package. Quantitative results were shown as mean±SD. The two-tailed Student's t test was used to calculate the statistical significance between groups. The chi-square test was used to analyze the relationship between IQGAP1 expression and clinicopathological characteristics. *P*<0.05 was considered statistically significant.

## Results

### Overexpression of IQGAP1 in ESCC

IQGAP1 has been implicated in many malignancies. In order to ascertain if expression of IQGAP1 is upregulated in ESCC tumor tissues, immunohistochemical analysis was performed on a TMA consisting of 75 paired ESCC tissue samples and adjacent normal tissues. As the results, the expression of IQGAP1 was observed in both cell membrane and cytoplasm (Figure 1A–C) which was consistent with previous studies [17]. For normal esophagus tissues, IQGAP1 protein was membrane staining and negative or weak cytoplasmic staining (Figure 1A). In contrast, the moderately or strongly cytoplasmic staining of IQGAP1 was detected at the tumor cells of ESCC tissues (Figure 1B–C). As summarized in Table 1, 92% (69/75) of ESCC tumors exhibited moderate and strong IQGAP1 cytoplasmic staining, and 8% (6/75) of ESCC tumors showed negative or weak IQGAP1 cytoplasmic staining. But only 29% (22/75) of normal adjacent tissues exhibited positive cytoplasmic staining for IQGAP1 protein. Statistical analysis indicated that IQGAP1 expression was upregulated in ESCC compared with adjacent normal tissue (*P*<0.0001).

**Figure 1:** Expression of IQGAP1 in ESCC and adjacent normal tissues. (A–C) Representative immunohistochemical staining of IQGAP1 expression in adjacent normal as well as ESCC tissue using TMA. IQGAP1 protein was membrane staining in normal esophagus tissues (A), moderate (B) and strong (C) cytoplasmic staining in ESCC tissues. (D) Western blot (Top) and RT-PCR (Bottom) demonstrated the IQGAP1 expression in ESCC tissues (T) and matched adjacent normal tissues (N) from four ESCC patients. β-actin or GAPDH was used as a loading control.

**Table 1:** The relationship between IQGAP1 expression and patient clinicopathologic characteristics

Variables	n	Negative n (%)	Positive n (%)	* *P*-value
Diagnosis				
Normal	75	53(71.0)	22(29.0)	**<0.0001**
Carcinoma	75	6(8.00)	69(92.0)	
Gender				
Male	55	5(9.00)	50(91.0)	NS
Female	20	1(5.00)	19(95.0)	
Age				
≤64	47	4(8.50)	43(91.5)	NS
>64	28	2(7.20)	26(92.8)	
T stage				
T1/T2	26	5(19.2)	21(80.8)	**0.03**
T3/T4	49	1(2.00)	48(98.0)	
Histologic grade				
Well and Moderate	57	4(7.00)	53(93.0)	NS
Poor	18	2(11.1)	16(88.9)	
Lymph node metastasis				
Negative	37	2(5.40)	35(94.6)	NS
Positive	38	4(10.5)	34(89.5)	
Distant metastasis				
Negative	70	6(8.60)	64(91.4)	NS
Positive	5	0(0.00)	5(100.0)	

*P-values were obtained by Chi-square test; ‘NS’ refers to ‘No statistical significance’.

To further analysis IQGAP1 expression in ESCC, Western blot analysis was performed in 4 paired primary ESCC tissues and adjacent normal tissues. The results revealed a significant elevation of IQGAP1 expression in tumors, as compared to the adjacent normal tissues (Figure 1D, top). In parallel with the upregulation of IQGAP1 protein, RT-PCR results showed that the mRNA level of IQGAP1 was also significantly upregulated in ESCC tissues compared with adjacent normal tissues (Figure 1D, bottom).

### Association between IQGAP1 expression and the clinicopathological features of ESCC

We further clarify the potential relationship between elevated expression of IQGAP1 and various clinicopathologic parameters. As shown in Table 1, elevated expression of IQGAP1 was significantly associated with pathologic T stage (*P*<0.05), and there was no significant association with gender, age, histologic grade, or lymph node and distant metastasis. These results support the notion that the increased IQGAP1 expression is associated with invasion depth of ESCC.

### Generation of stable IQGAP1 silencing clones in ESCC cell lines

To further investigate the role of IQGAP1 in ESCC cell lines, the IQGAP1 protein level in KYSE150 and EC9706 cell lines was determined. Western blot analysis revealed that IQGAP1 protein was highly expressed in EC9706 and KYSE150 cells compared with normal esophageal cell line (Het-1A) (Figure 2A).

**Figure 2:** Expression of IQGAP1 in ESCC cell lines and establishment of IQGAP1 knockdown stable cell lines. (A) Western blots showing the expression of IQGAP1 in Het-1A, KYSE150 and EC9706 cell lines. (B) EC9706 or KYSE150 cells were stable transfected with control or IQGAP1-shRNA vector, and IQGAP1 protein and mRNA expression in control and IQGAP1 knockdown stable cell lines were assessed by Western blot and RT-PCR. (C) Western blot analysis of the expression of IQGAP1 in two EC9706/IQGAP1 (E1 and E2) or KYSE150/IQGAP1 (K1 and K2) knockdown stable clones and one vector control clone (EC9706/control or KYSE150/control). (D) The histogram represents quantitative densitometry of proteins of the results of 3 independent experiments (mean±SD). *, Statistically different, compared with the control cells (*P*<0.05).

To study the function of IQGAP1 gene in ESCC cells, knockdown of IQGAP1 was achieved by stable transfecting EC9706 and KYSE150 cells with IQGAP1-targeted RNAi expression vectors (IQGAP1-shRNA) or a control vector. After selecting with G418, several independent stable clones were isolated and the stable silencing effect of IQGAP1 was identified by Western blot and RT-PCR. The results showed that the levels of both IQGAP1 protein and mRNA were significantly reduced in either EC9706 or KYSE150 cells transfected with IQGAP1-shRNA compared to those with the control vector (Figure 2B). Two IQGAP1 knockdown stable clones in EC9706 (E1 and E2 clones) or KYSE150 cells (K1 and K2 clones) and corresponding one vector control clone (EC9706/control or KYSE150/control clone) were selected for further analysis (Figure 2C). The protein quantification showed that IQGAP1 expression level was efficiently reduced by 80% in EC9706/IQGAP1 knockdown clones and 70% in KYSE150/IQGAP1 knockdown clones compared with control clone (Figure 2D).

### Suppression of IQGAP1 expression in ESCC cells inhibits cell growth

To test the effect of IQGAP1 knockdown on ESCC cell growth, MTT assay was performed and growth curves were generated. As shown in Figure 3A and B, cell proliferation was remarkably inhibited in IQGAP1 knockdown clones when compared with control clone (*P*<0.05). In addition, the colony formation assay further revealed effects of IQGAP1 knockdown on growth properties of ESCC cells. The numbers of colonies had an average 3–5 folds decrease in IQGAP1 knockdown clones compared with the control clone (*P*<0.05; Figure 3C–D). Moreover, the colonies from control cells were much larger than those from the IQGAP1 knockdown stable cells (Figure 3C). Overall, the dramatic reduction of growth and colony formation of IQGAP1 silenced cells suggest that IQGAP1 suppression may negatively regulate ESCC cell growth.

**Figure 3:** Knockdown of IQGAP1 expression inhibits proliferation of ESCC cells. (A–B) MTT proliferation assay. Equal numbers of cells were cultured and monitored for growth over time. Each graph indicates the average number of viable cells assessed at 2, 4, 6, 8 or 10 days. The data shown represent mean±SD from three independent experiments. (C) Representative images of the colony formation assay were shown. (D) The histogram represents number of colonies of the results of 3 independent experiments (mean±SD). *, Statistically different, compared with the control cells (*P*<0.05).

### Suppression of IQGAP1 expression in ESCC cells inhibits cell cycle progression

To investigate the mechanism of IQGAP1 knockdown inhibiting cell proliferation, flow cytometry was performed to determine the cell cycle distribution. Compared with control cells, IQGAP1 knockdown cells displayed a significant increase in G0/G1 phase (*P*<0.05; Figure 4A). Consistent with previous studies [22], we further found that IQGAP1 knockdown significantly downregulated expressions of cyclin D1 and CDK4 which are related to the G1 progression and G1/S transition of the cell cycle, while it had no significant effect on the levels of cyclin B1 and CDK1 which are related to the G2/M phase transition (Figure 4B). These results suggest that reduction in IQGAP1 expression in EC9706 and KYSE150 cells by RNAi induces cell cycle arrest in the G1 phase and suppresses ESCC cell proliferation.

**Figure 4:** Knockdown of IQGAP1 expression inhibits cell cycle progression. (A) The cells were fixed and stained with propidium iodide and the cell cycle was analyzed by flow cytometry. The percentage of cells in different cell cycle phase is shown as the mean±SD of 3 independent experiments. *, Statistically different, compared with the control cells (*P*<0.05). (B) Protein expression levels of cyclin D1, CDK4, cyclin B1 and CDK1 were examined by Western blot.

### Suppression of IQGAP1 expression inhibits migration and invasion of ESCC cells *in vitro*

Tumor cell migration and invasion are two critical steps in cancer metastatic process. We investigated cell migration by wound healing assay and non-matrigel-coated Boyden chamber. As shown in Figure 5A, although the EC9706/control cells migrated rapidly into the wound area to cause most of wound closure within 48 h, a significant wound closure inhibition was observed in the EC9706/IQGAP1 knockdown cells. Similarly, the KYSE150/control cells were completely distributed at the wound area within the 48 h incubation, whereas the KYSE150/IQGAP1 knockdown cells exhibited delayed closure of the wound (Figure 5A). The cellular migrations were decreased 5–8 folds in IQGAP1 knockdown cells at 48 h compared with control cells (*P*<0.05; Figure 5B–C). We further carried out transwell assay to determine the cell migration ability. Compared with control cells, IQGAP1 knockdown in EC9706 or KYSE150 cells displayed a marked decrease in number of cells across the transwell membrane (Figure 5D–E). The number of IQGAP1 knockdown cells that passed through the membrane was decreased 9-fold compared with that of control cells (*P*<0.05; Figure 5F). Taken together, suppression of IQGAP1 expression may decrease *in vitro* migration of ESCC cells.

**Figure 5:** Knockdown of IQGAP1 expression inhibits the migration and invasion of ESCC cells *in vitro*. (A) Wound healing assays. The confluent monolayer of cells was wounded and photographed at the indicated time points. (B–C) The distances covered by the cells (wound width) were plotted in term of pixels. The data shown represent mean±SD of 3 independent experiments. *, Statistically different, compared with the control cells (*P*<0.05). Representative microscopy images of the migration and invasion assays in EC9706 (D) and KYSE150 (E) cells. The cell number quantifications of cell migration (F) and invasion (G) represent mean±SD of 3 independent experiments. *, Statistically different, compared with the control cells (*P*<0.05).

We further investigated cell invasion by matrigel-coated invasion chamber assays. As shown in Figure 5D and E, IQGAP1 knockdown in EC9706 and KYSE150 cells also markedly reduced cell invasion properties when compared to control cells. There was a 10-fold decrease in invasiveness of the IQGAP1 knockdown cells compared with the control cells (*P*<0.05; Figure 5G). This finding indicates that suppression of IQGAP1 expression can inhibit *in vitro* invasion of ESCC cells.

### Suppression of IQGAP1 expression decreases the growth and metastasis of tumor cells *in vivo*

Subcutaneous tumor growth assays in nude mice were performed to investigate the effect of IQGAP1 knockdown on tumor growth in *vivo*. The tumors formed by control cells grew faster than the IQGAP1 knockdown ones (*P*<0.05; Figure 6A). All mice were sacrificed 12 weeks after injection, and the final tumor volumes in IQGAP1 knockdown groups were markedly smaller than those in control group (Figure 6B). These results indicate that knockdown of IQGAP1 expression in ESCC cells can suppress *in vivo* tumor growth.

**Figure 6:** Knockdown of IQGAP1 expression reduces tumor growth, invasion and metastases *in vivo*. (A) The curve showed that the tumor growth of IQGAP1 knockdown groups in EC9706 or KYSE150 cells was significantly inhibited compared to that of control group. The data shown represent mean±SD, n = 6 animals/group. (B) Representative images showed that the tumor size of IQGAP1 knockdown groups in EC9706 or KYSE150 was markedly smaller on the 12 week after tumor cells inoculation than that of control group. Mice were killed 12 weeks after injection, and lungs were excised and photographed (C), and 4-µm paraffin slices of tumor (D), lymph node (E) and lung (F) tissues were stained with H&E dyes and examined under a light microscope. Arrows indicate the presence of invasional striated muscle in tumor slice and a metastatic tumor in lung slice. Magnification, ×100.

Given that increased cell migration and invasion contribute to the metastatic potential of cancer cells, we tested whether suppression of IQGAP1 expression would affect the invasive and metastatic ability of ESCC cells *in vivo*. In EC9706/control (or KYSE150/control) group, cancer cells extensively invaded surrounding muscle tissues in 4 (or 6) mice. In contrast, in IQGAP1 knockdown groups, no obvious invasion of tumor cell into surrounding muscle tissues was found, and tumor lesions were apparently separated from surrounding muscle tissues (Figure 6D). These data indicated that the invasion ability of cancer cells was attenuated by knockdown of IQGAP1 expression. Further, 3 (or 2) mice developed lymph node metastases in EC9706/control (or KYSE150/control) group (Figure 6E), whereas in IQGAP1 knockdown groups, no gross or microscopic lymph nodes were observed, which showed that the incidence of lymph node metastasis were significantly inhibited by downregulation of IQGAP1 expression. In addition, 3 mice developed visually observable metastatic lung nodules and 2 mice developed small tumor nodules that were detected only by staining lung sections with H&E in EC9706/control group. However, only 1 small tumor nodule was found under the microscope in H&E sections of mouse lungs in the EC9706/IQGAP1 knockdown groups. Representative lungs and their corresponding H&E staining were shown in Figure 6C and F. These results showed that the incidence of lung metastasis was significantly attenuated by knockdown of IQGAP1 expression. No metastatic tumor was found in lungs of all KYSE150 groups (Figure 6C and F). These data suggest that knockdown of IQGAP1 expression has the potential to inhibit tumor invasion and metastases *in vivo*.

### IQGAP1 knockdown reverses epithelial to mesenchymal transition (EMT)

EMT of cancer cells is an early event leading to local invasion and metastasis to a new location. To determine whether the IQGAP1 involved in EMT process, we examined the expressions of EMT epithelial maker E-cadherin and mesenchymal maker N-cadherin in IQGAP1 knockdown and control cells. Results of Western blot indicated that IQGAP1 knockdown caused an increase in the levels of E-cadherin with a concomitant downregulation of N-cadherin (Figure 7A). These results were further confirmed by immunofluorescence experiments (Figure 7B) which showed that the expression of E-cadherin was increased, whereas that of N-cadherin was decreased in IQGAP1 knockdown cells. The immunofluorescence also confirmed that IQGAP1 expression was depleted by the specific knockdown in EC9706 and KYSE150 cells. These data suggest that IQGAP1 might play an important role in promoting the EMT process.

**Figure 7:** Effect of IQGAP1 knockdown on the expression of epithelial and mesenchymal markers. (A) Western blot analysis of E-cadherin and N-cadherin in IQGAP1 knockdown and control cells. (B) Immunofluorescence microscopy analysis of IQGAP1, E-cadherin and N-cadherin in IQGAP1 knockdown and control cells. The red signal represents the staining of corresponding protein, and the blue signal represents the nuclear DNA staining by DAPI.

## Discussion

Recently, increasing evidence reveals that IQGAP1 plays an important role in biological processes of many cancers. Nevertheless, the exact role of IQGAP1 in tumor progression is not unclear, and the function of IQGAP1 in tumor cell biology of ESCC has not been thoroughly investigated. To address these issues, we first investigated the expression of IQGAP1 in ESCC clinical samples by immunohistochemistry, Western blotting and RT-PCR. Different methods showed similar results. Our results clearly showed that IQGAP1 was upregulated at both the mRNA and protein levels in ESCC tissue. The immunohistochemical analysis on TMA showed that IQGAP1 was overexpressed in 92.0% (69/75) ESCC specimens, whereas weak or no IQGAP1 expression in adjacent normal tissues. Statistical analysis revealed that IQGAP1 expression significantly correlated with invasion depth of ESCC. The previous reports have demonstrated that IQGAP1 is overexpressed in several malignancies. Furthermore, IQGAP1 expression has been noted to be associated with more aggressive behavior [21]. Our studies are consistent with these observations, which support our proposal that IQGAP1 may play critical roles in the initiation and progression of ESCC. The aberrant overexpression of IQGAP1 in ESCC may make it a good candidate as a therapeutic molecular target.

To further investigate the biological role of IQGAP1 expression in ESCC progression, we have used a short hairpin RNAi technique to stably suppress IQGAP1 expression in two ESCC cell lines, EC9706 and KYSE150 cells, with high level of IQGAP1 expression. IQGAP1 has been successfully downregulated by RNAi in some previous studies [10]–[11], [23], but the downregulation of IQGAP1 expression by RNAi in ESCC cells has not been performed until now. As shown here, shRNA targeting IQGAP1 resulted in the efficient and specific downregulation of IQGAP1 protein and mRNA. Significantly, IQGAP1 knockdown not only inhibited tumor cell proliferation by arresting the cells in the G1 phase of the cell cycle, as well as migratory and invasive activities *in vitro*, but also significantly diminished tumor growth, invasion and lymph node and lung metastatic ability *in vivo* using a xenograft model. In order to rule out the possible off-target effects, we utilized stable transfection of another shRNA (IQ-sh) targeted to different regions of IQGAP1 mRNA to silence for endogenous IQGAP1 in EC9706 and KYSE150. The data demonstrated that stable suppression of IQGAP1 expression was able to reduce cell proliferation and invasion capability *in vitro* (Figure S1) which were consistent with observations from stable transfection IQGAP1-shRNA. Recently, evidence also indicates that increasing IQGAP1 expression in breast cancer MCF-7 cells promotes cell proliferation and invasion [23], siRNA-induced knockdown of IQGAP1 reduces the proliferation and invasion of thyroid cancer [10] and MCF-7 cells [23]. To our knowledge this is the first report on the direct effect of IQGAP1 siRNA on ESCC cell proliferation and metastasis. Our studies are directed at understanding the potential role of IQGAP1 in the behavior of malignant ESCC cells. Therefore, these results indicate a possible role for IQGAP1 in malignancy progression of ESCC and IQGAP1-siRNA can be used as a novel drug for therapeutic targeting of IQGAP1 in ESCC.

EMT is such process which allows epithelial cells to change their phenotype, acquire mesenchymal properties, and increase their capability to migrate [24]. Accumulating evidence has shown that EMT plays an important role in cancer progression and metastasis [25]. Molecular hallmarks of EMT include down-regulation of E-cadherin, which is responsible for the loss of cell-cell adhesion; upregulation of mesenchymal-related proteins N-cadherin, which mediates cell-cell adhesion and modulates cell migration and tumor invasiveness [26]. Interestingly, here we showed that downregulation of IQGAP1 led to a reversion of EMT progress, characterized by decreased expression of mesenchymal markers N-catenin and increased expression of epithelial markers E-cadherin, which was in agreement with IQGAP1 knockdown inhibiting invasion and metastasis of ESCC cell lines *in vitro* and *in vivo*. Indeed, it has been found that IQGAP1 binds directly to E-cadherin and overexpression of IQGAP1 reduces E-cadherin-mediated adhesion and facilitates cancer cells to metastasize [27]. These findings present a pivotal role of IQGAP1 in EMT process and tumor promoting function in metastasis of ESCC. IQGAP1, as a scaffold protein, contributes to the transformed cancer cell phenotype by regulating several distinct signaling pathways. Therefore, further research needs to be conducted in order to determine new target protein and molecular mechanism of IQGAP1 contributing ESCC development.

In conclusion, our data have provided evidence that IQGAP1 expression is unregulated and correlated with the invasion depth of ESCC. Importantly, by using RNAi technology we have successfully silenced IQGAP1 gene in EC9706 and KYSE150 cells, and for the first time found that downregulation of IQGAP1 expression could inhibit the growth and metastasis of ESCC cells *in vitro* and *in vivo*. Further, downregulation of IQGAP1 may lead to a reversion of EMT progress. Therefore, the findings in this study present new insights into the potential role of IQGAP1 in ESCC occurrence and progression, and targeted knockdown of IQGAP1 may represent a promising approach for ESCC treatment.

## Supporting Information

Figure S1 **The effects of stable suppression of IQGAP1 expression on ESCC cell proliferation and invasion** ***in vitro*** **.** (A) EC9706 or KYSE150 cells were stably transfected with IQ-sh vector, and IQGAP1 protein expression in two stable clones was assessed by Western blot. (B) Cell numbers were measured at 2–10 days by MTT assay. (C) Transwell invasion assay of EC9706 and KYSE150 cells after IQGAP1 downregulation. (D) Quantitative analysis of the number of invasive cells. Results are mean±SD of 3 independent experiments. *, Statistically different, compared with the control cells (*P*<0.05).
(TIF)
